# The Antibacterial Activity of Chitosan Products Blended with Monoterpenes and Their Biofilms against Plant Pathogenic Bacteria

**DOI:** 10.1155/2016/1796256

**Published:** 2016-04-04

**Authors:** Mohamed E. I. Badawy, Entsar I. Rabea, Nehad E. M. Taktak, Mahmoud A. M. El-Nouby

**Affiliations:** ^1^Department of Pesticide Chemistry and Technology, Faculty of Agriculture, Alexandria University, El-Shatby, Alexandria 21545, Egypt; ^2^Department of Plant Protection, Faculty of Agriculture, Damanhour University, Damanhour 22516, Egypt; ^3^Department of Tropical Health, High Institute of Public Health, Alexandria University, Alexandria 21561, Egypt

## Abstract

This study focuses on the biological activities of eleven chitosan products with a viscosity-average molecular weight ranging from 22 to 846 kDa in combination with the most active monoterpenes (geraniol and thymol), out of 10 tested, against four plant pathogenic bacteria,* Agrobacterium tumefaciens*,* Erwinia carotovora*,* Corynebacterium fascians*, and* Pseudomonas solanacearum*. The antibacterial activity was evaluated* in vitro* by the agar dilution technique as a minimum inhibitory concentration (MIC) that was found to be dependent on the type of the microorganism tested. The most active product of chitosan was used for biofilm production enriched with geraniol and thymol (0.1 and 0.5%) and the films were also evaluated against the tested bacteria. The biological bioactivities summarized here may provide novel insights into the functions of chitosan and some monoterpenes and potentially allow their use for food protection from microbial attack.

## 1. Introduction

Foodborne pathogens are a major concern for consumers, the food industry, and food safety authorities. In recent years, considerable effort has been made to find natural antimicrobials that can inhibit bacterial and fungal growth in foods in order to improve their quality and shelf life. Similarly, consumers have become concerned about the safety of synthetic preservatives that are used in foods. Biopolymer chitosan and its derivatives are very attractive for agricultural applications as they are safe to human and environment. Due to their high biological activity, biodegradability, biocompatibility, and nontoxicity to mammals and nontarget organisms, chitosan products are recently widely used as biocides either alone or blended with other natural products [1–4]. Chitosan is a linear copolymer of glucosamine (GlcN) and* N*-acetylglucosamine (GlcNAc) units linked by 1,4-glycosidic bonds and is obtained through the alkaline hydrolysis of chitin [5, 6]. The antimicrobial activity of chitosan is influenced by many factors, such as its concentration [7, 8], degree of polymerization (DP) or molecular weight (MW) [9, 10], degree of acetylation (DA) [11], pH, and ionic strength of the media [12] as well as the biological sources of chitosan [13]. Many studies performed on the effect of the MW of chitosan molecule on the antimicrobial activity have shown diverging results. While some studies confirmed that the high MW chitosan had higher antimicrobial activity than the low MW chitosan [14, 15], other studies reported opposite results [16, 17]. However, as most research studies involved chitosan with only one or very few different MWs that were not obtained from the same source or by the same method, these data may not give comparable results [4, 18, 19].

In plant pathology, the antimicrobial activities of chitosan compounds have been mainly evaluated on plant fungal pathogens [20–23], and few studies were done on chitosan action directed towards viruses and bacteria in plant [24–26]. From the literature, it can be noted that the antibacterial activity of chitosan has been widely studied against food and clinically important bacteria; however, this fact has not been matched with plant pathogenic bacteria [27].

Monoterpenes are a class of terpenes that consist of two isoprene units and have the molecular formula C_10_H_16_. Monoterpenes may be linear (acyclic) or may contain rings. The antimicrobial activity of monoterpenes was recognized long ago, but their application as natural antimicrobials has recently received increased attention in the food industry [7, 28, 29]. The high antimicrobial activity of some monoterpenes against many agricultural pathogens such as bacteria and fungi makes these products useful as potential alternatives to harmful synthetic pesticides as well as good lead compounds for the development of safe, effective, and fully biodegradable pesticides [7, 30, 31]. Many studies proved that the incorporation of biologically active components such as plant essential oils that contain monoterpenes into chitosan films not only may enhance the antimicrobial properties of the films but also can reduce water vapor permeability and slow lipid oxidation of the product on which the film is applied [28, 32, 33].

Therefore, the objectives of the present work were (1) to study the antibacterial activity of chitosan products with different MWs and their blends with geraniol and thymol as the most active monoterpenes against four crop-threatening bacteria,* Agrobacterium tumefaciens*,* Erwinia carotovora*,* Corynebacterium fascians*, and* Pseudomonas solanacearum*, (2) to study the preparation and antibacterial assay of different chitosan films by microdilution nutrient broth spectrophotometric technique, and (3) to study the antibacterial activity of monoterpenes incorporated into chitosan films by inhibition zone technique. The data aims to use well-defined chitosan with respect to MW and to determine which chitosan film shows the greatest inhibitory effect against the most common plant pathogens.

## 2. Materials and Methods

### 2.1. Chemicals and Plant Pathogenic Bacteria

Eleven chitosan products with a viscosity-average molecular weight ranging from 22 to 846 kDa previously produced from shrimp shells according to Badawy and coauthors were used in this study [34]. Geraniol (98%), thymol (98%), 2,3,5,-triphenyltetrazolium chloride (TTC), and* N*,*N*-dimethyl-1,4-phenylenediamine (DMPD) were purchased from Sigma-Aldrich Co. (USA). Nutrient agar (NA) was purchased from Oxoid Ltd. (Basingstoke, Hampshire, UK). Nutrient broth (NB) medium was used to grow the bacterial strains to a final inoculum size of 5 × 10^5^ CFU/mL. All of the other reagents used were of high purity grade. Microorganisms used in this work were four bacteria:* Agrobacterium tumefaciens*,* Erwinia carotovora*,* Corynebacterium fascians*, and* Pseudomonas solanacearum* (Microbiology Laboratory, Department of Plant Pathology, Faculty of Agriculture, Alexandria University, Egypt). Bacteria were maintained on NA medium at 37 ± 2°C.

### 2.2. Preparation of Chitosan Composite Films

A series of active composite biopolymers films were prepared by casting the composite polymers (chitosan with gelatin or starch) with different concentrations of glycerol and sorbitol (1, 2, 5, and 10%, w/w) as plasticizers. The best film was selected to immobilize it with the most active monoterpenes (geraniol and thymol) as follows. Chitosan stock solution (2%, w/v) was prepared in 1% (v/v) aqueous acetic acid solution. Geraniol and thymol were dissolved in DMSO and then mixed with Tween 20 (Aldrich Chemical Co.) to help distribute and completely incorporate the compound in chitosan matrix and then added to the chitosan stock solution. The final film forming solution consisted of 2% chitosan, 1% acetic acid, 2% starch, 1% sorbitol as a plasticizer, 0.05% Tween 20, and 0.1% or 0.5% geraniol or thymol. The mixture was stirred for homogenization under aseptic conditions for 1 min and poured into 50 mm inner diameter sterile Petri dishes. All the films were prepared with 5 g of film solution per Petri dish (1 film), which ensured 20 mg chitosan/film. Control films were prepared identically but without addition of monoterpenes. After drying at 25°C and 50% relative humidity for 72 h, films were manually peeled off and then kept in sealed Petri dishes at 4°C until being used [35].

### 2.3. Characterizations of the Chitosan Films

#### 2.3.1. Film Thickness

Film thickness was measured with a precision digital low-pressure micrometer (6-inch LCD Digital Vernier Caliper/Micrometer Gauge 150 mm, Shenzhen, China) with an accuracy of ±0.02 mm/0.001 inches. Five thickness values were taken at five random locations on the films. Mean thickness values for each sample were calculated and used in water vapor permeability (WVP) calculation.

#### 2.3.2. Microstructural Analysis

Scanning electron microscope (SEM) analyses were useful to indicate the microstructural analysis of the film surface and give an insight into system microstructure. The measurements were performed using a JEOL JSM-5410 (Japan) electron microscope. Pieces of 5 × 1 mm^2^ were cut from the films and mounted in copper stubs. Samples were gold coated and observed using an accelerating voltage of 10 kV. Photographs were taken at magnification ×10000 for surface morphologies and ×2000 for their cross section.

#### 2.3.3. Water Vapor Permeability (WVP)

WVP of each film was determined using the gravimetric Modified Cup Method based on ASTM method [36] and adapted to hydrophilic edible films by McHugh and coauthors [37]. The circular test vials made of glass with 15 mm internal diameter and 60 mm height were filled with 10 g of silica gel (desiccant) to produce a 0% RH. Films without pinholes or any defects were sealed to the vial mouth containing silica gel. After taking the initial weight of the test vials, the vials were kept in a desiccator with 90 ± 5% RH maintained with a saturated sodium chloride solution (26%, w/v) at 25° ± 2°C. Weight gain measurements were taken by weighing the test vial with an analytical balance (±0.0001 g) every day for one week. A plot of weight gained versus time was used to determine the water vapor transmission rate (WVTR). The slope of the linear portion of this plot represented the steady state amount of water vapor diffusing through the film per unit time. The WVTR was expressed as gram units, per square meter, per day (g/m^2^·d), which was calculated from the slope of the straight line and then divided by the exposed film area (m^2^). The WVP of the films was then calculated by multiplying the WVTR by the film thickness (mm). Three samples per each film were tested.

#### 2.3.4. Swelling Index

The swelling index of the prepared films was estimated as follows: chitosan blend films were cut by cork borer with diameter 0.8 mm and dried in oven for 20 min at 60°C. The films were weighed and then immersed in distilled deionized water (10 mL per each film in glass vial) and allowed to swell and reach the equilibrium for 24 h at 25°C. After different time intervals (0.5, 2.5, 4, and 24 h), the excess surface water on the film was removed by being wiped with soft paper and water gain of the films was weighed. The content of water absorbed in chitosan films as swelling index was calculated as follows:

(1) $$\begin{array}{c} \text{Swelling index}=\left[\;\frac{\left(W_{t}-W_{o}\right)}{W_{o}}\;\right], \end{array}$$

where *W*_*t*_ and *W*_*o*_ are the weights of swollen film at time *t* and that of the original film weight, respectively. Experiments were performed in triplicate, and the data obtained were averaged.

#### 2.3.5. Antioxidant Activity

The antioxidant activity of the films was determined according to the method described previously by Fogliano and coauthors [38] with some modifications. DMPD (100 mM) was prepared and 1 mL of this solution was added to 100 mL of 100 mM acetate buffer, pH 5.25, and the coloured radical cation (DMPD^+^) was obtained by adding 0.2 mL of a 50 mM solution of ferric chloride (the final concentration was 0.1 mM). 2 mL of this solution was transferred directly to the plastic cuvette (10 mm in length) and its absorbance at 505 nm was measured (*t*_0_) using a UV-visible spectrophotometer (Alpha-1502 UV-Visible Spectrophotometer, LAXCO, Inc., Bothell, Washington, USA). An optical density of 0.900 ± 0.100 unit of absorbance was obtained and it represents the uninhibited signal at time *t*_0_. The films were cut into small pieces (10 mg) and immersed in 2 mL of coloured radical cation (DMPD^+^) solution (0.1 mM) and incubated for 10 min with shaking at room temperature in the dark. After this time, a decrease in absorbance was measured (*t*_10_) and the results were expressed as mg equivalents of ascorbic acid equivalent per g of film, based on standard curves previously prepared for ascorbic acid. The test was carried out in triplicate.

### 2.4. The* In Vitro* Antibacterial Assay

#### 2.4.1. The Antibacterial Assay of Chitosan Compounds and Their Blends with Geraniol and Thymol

The* in vitro* antibacterial activity of chitosan, geraniol, and thymol compounds was assayed using NA dilution method according to the European Committee for Antimicrobial Susceptibility Testing (EUCAST) [39] against* A. tumefaciens*,* E. carotovora*,* C. fascians*, and* P. solanacearum*. The chitosan compounds were dissolved in 0.5% (v/v) aqueous acetic acid and diluted to obtain the required stock. The pH of the chitosan solutions was adjusted to 5.5–6.0 with 1 M NaOH. Geraniol and thymol were dissolved in dimethyl sulfoxide (DMSO) to obtain the main stock solution. For determination of MIC, different concentrations of chitosan (100–3000 mg/L) and geraniol and thymol (10–2000 mg/L) were added to NA medium immediately before it was poured into the Petri dishes at a temperature of 40–45°C. Parallel controls were maintained with distilled water, aqueous acetic acid (0.5%, v/v), and DMSO mixed with NA medium. One loopful of microorganism suspensions in NB medium (≈6 *μ*L) was spotted on the surface of NA medium (ten spots per plate) and then incubated at 37 ± 2°C for 24 h. Each concentration was tested in triplicate. The MIC was recorded in each case as the minimum concentration that inhibited the growth of the tested microorganism after the incubation period. From the MIC observed, the intermediate concentrations between MIC values were prepared by suitable dilution of stock solution and the accurate MIC values were determined.

#### 2.4.2. The Antibacterial Assay of Chitosan Films by NB Spectrophotometric Technique

The bacterial growth inhibition by chitosan films was spectrophotometrically measured by using TTC as a chromogenic marker [40] with some modifications. A fixed weight of each film (0.005 g) was immersed into sterile tube which contains 4 mL of NB medium and 50 *μ*L of each bacterial suspension (5 × 10^5^ CFU/mL). The tubes were mixed on a microplate shaker at 200 rpm for 1 min prior to incubation for 24 h at 37 ± 2°C. Controls were prepared with culture medium, bacterial suspension only. To indicate respiratory activity, 200 *μ*L of each tube was added to the wells of a sterile 96-well microtitre plate, with the addition of 20 *μ*L/well of TTC dissolved in water (0.01%, w/v), and incubated under appropriate cultivation conditions for 30 min in the dark. The absorbance was measured at 492 nm in an Ultra Microplate Reader (Robonik, Pvt. Ltd.). Positive controls were wells with a bacterial suspension. Negative controls were tubes with growth medium and the tested compounds. The bacterial growth inhibition percentage was calculated on the basis of the metabolic activity.

#### 2.4.3. The Antibacterial Assay of Chitosan Films by Inhibition Zone Technique

50 *μ*L of bacterial colony suspension of each bacterium containing 5 × 10^5^ CFU/mL of NB medium was dropped at the center of the sterile Petri dish containing NA (yeast extract, peptone, glucose, and agar) and mixed well. After diffusion of the bacterial suspension in the medium, uniform 10 mm diameter discs of the chitosan film were cut with a hole-puncher (10 mm in diameter) from the prepared chitosan films, and 1 film disc was placed in the center of the inoculated Petri dish. Chitosan films with no monoterpenes served as control. The plates were incubated at 37°C, and measurements were taken after 48 h. During the incubation, the film discs slightly swelled due to water absorption and resulted in enlarged diameter; therefore, both the inhibition zone surrounding the discs and the disc diameter were measured, and the width of the inhibition ring was recorded. The tests were performed in triplicate.

### 2.5. Statistical Analysis

Statistical analysis was performed using the SPSS 21.0 software (Statistical Package for Social Sciences, USA). Analysis of variance (ANOVA) of the data was conducted and means property values were separated (*P* ≤ 0.05) with Student-Newman-Keuls (SNK) test for the property values. Differences were considered significant at *P* ≤ 0.05.

## 3. Results and Discussion

### 3.1. The Antibacterial Activity of Chitosan Products and Their Blends with Geraniol and Thymol

The antibacterial activities of different-molecular-weights chitosan (22 to 846 kDa) alone or in combination with geraniol and thymol against* A. tumefaciens*,* C. fascians*,* E. carotovora*, and* P. solanacearum* are shown in Table 1 as MIC values. The result showed that the MW of chitosan plays an important role in the biological activity wherein its increase, the antibacterial activity, has been reduced. The strongest antibacterial activity was exhibited by chitosan of 22 kDa (Ch1) against the four kinds of bacteria tested with MIC 800, 900, 850, and 600 mg/L against* A. tumefaciens*,* C. fascians*,* E. carotovora*, and* P. solanacearum*, respectively. However, Ch11 (MW 846 kDa) revealed the lowest inhibitory effect among the products with MIC 1300, 2600, 2100, and 1225 mg/L against* A. tumefaciens*,* C. fascians*,* E. carotovora*, and* P. solanacearum*, respectively.

As geraniol and thymol exhibited the highest antibacterial activity, among different monoterpenes, against these tested bacteria (data not shown), the effect of blending chitosan compounds with both monoterpenes at different concentrations was tested and the data are shown in Table 1. The data against* A. tumefaciens* indicate that the mixture of 500 mg/L of each chitosan compound with different concentrations of geraniol proved MICs ranged from 220 to 500 mg/L. There are no clear differences between the activities of the mixtures of chitosan compounds (Ch1–Ch10) with geraniol; however, the mixture of Ch11 + geraniol was significantly the lowest active (MIC = 500 mg/L). Blending of chitosan compounds with thymol enhanced the antibacterial activity compared to geraniol and the most potent blend was Ch7 (241 kDa) + thymol with MIC 75 mg/L. The antibacterial activity against* C. fascians* showed that the highest activity was obtained with the mixtures of Ch3 (64 kDa) + geraniol and Ch3 + thymol with MICs = 170 and 25 mg/L, respectively. The results also proved that the chitosan-thymol mixtures showed the highest inhibition activity against* C. fascians* compared to the other tested bacteria. The antibacterial activity against* E. carotovora* shows that the highest activity was also obtained with the mixtures of Ch3 + geraniol and Ch3 + thymol with MICs = 210 and 40 mg/L, respectively. However, there is no clear difference between the activities of the mixtures of chitosan compounds (Ch1–Ch10) with geraniol. The data against* P. solanacearum* show that the mixture of 500 mg/L of each chitosan compound with different concentrations of geraniol resulted in MICs ranging from 250 to 375 mg/L with no clear differences between the tested chitosan compounds (Ch1–Ch11) with geraniol. However, the inhibition activity was significantly enhanced when thymol was added to the chitosan compounds with MICs from 50 mg/L (Ch6 + thymol) to 140 mg/L (Ch11 + thymol).

The MW of chitosan products plays an important role in biological activity; however, there is no clear correlation between the MW and the antimicrobial activity. The differences between the obtained data in many research studies may result from the different DDA, DP, and MW distributions of chitosan [1]. The antibacterial activity of three-MW chitosan products (360, 611, and 953 kDa) was tested* in vitro* against* A. tumefaciens*,* C. fascians*,* E. amylovora*,* E. carotovora*,* P. solanacearum*, and* S. lutea* [41]. The results indicated that chitosan had a direct effect on bacterial cells and the activity increased with the increase of the MW up to MIC 500 mg/L for* C. fascians*. In contrast, another three-MW chitosans (5, 37, and 57 kDa), prepared from a commercial product of 290 kDa, showed that the lowest MW (5 kDa) exhibited the highest activity against* A. tumefaciens* (MIC = 2600 mg/L), while chitosan 37 kDa was the most active against* E. carotovora* (MIC = 950 mg/L) [42]. The activity in the present study was increased with the decrease in the MW that was in agreement with previous studies that reported that oligochitosan which was produced from chitosan hydrolysis not only was water soluble but also was more effective than native chitosan [16, 43]. Another study demonstrated that MW chitosans (≤10 kDa) have greater antibacterial activity than high MW chitosans [44]. Chitosan and monoterpenes as natural polymers have great potential for usage in bio-based packaging materials. The current study showed that the incorporation of monoterpenes into chitosan films improved the antibacterial and antioxidant properties.

### 3.2. Characteristics of the Chitosan Films

Different chitosan biofilms (32 films) with different ratios of each component (chitosan (2%), gelatin or starch (2 and 5% of each), and plasticizers (glycerol or sorbitol)) at 1, 2, 5, and 10% were prepared. The films were divided into four groups as follows: GI (chitosan + gelatin + glycerol), GII (chitosan + gelatin + sorbitol), GIII (chitosan + starch + glycerol), and GIV (chitosan + starch + sorbitol). The best film in performance was selected to be used for incorporation of the most biologically active monoterpenes (geraniol and thymol) as antimicrobial film. This biofilm consists of chitosan (2%), starch (2%), and sorbitol (1%).

The physicochemical properties (dry weight, thickness, WVP, antioxidant activity, and swelling index) of the modified chitosan film with geraniol and thymol are illustrated in Table 2. Dry weight, thickness, and antioxidant properties were improved largely after incorporating geraniol and thymol into chitosan film. There is a significant difference between the film without monoterpenes (Ch/starch) and that incorporated with geraniol and thymol. The dry weight increased from 0.150 g (Ch/starch) to 0.231 g (Ch/starch + 5% Thymol). However, there were no significant differences between the four specimens incorporated with geraniol and thymol. The same trend was found with the thickness of the films where the films which have different concentrations of geraniol or thymol were different significantly with Ch/starch (0.068 mm). The highest thickness (0.124 mm) was recorded with Ch/starch-thymol composite film at 0.5%. Films with 0.1% or 0.5% geraniol increased the WVP (48.88 and 70.49 g/m^2^·d, resp.) compared to 40.12 g/m^2^·d for Ch/starch alone. However, the Ch/starch film incorporated with thymol (0.1 and 0.5%) significantly reduced the WVP (36.48 and 29.76 g/m^2^·d, resp.). This finding is based on the use of the possibility of such postharvest film coatings for perishable agricultural products and can slow down the oxidation of lipids on which the film is applied as the decrease of the WVP.

The antioxidant activity of the films has been expressed as mg equivalents of ascorbic acid equivalent per g of film. All chitosan films showed antioxidant activity and there is no significant difference between all films (Table 2). Ch/starch film with thymol gave higher antioxidant activity than Ch/starch film with geraniol and the antioxidant activity is concentration-dependent.

In an attempt to study the microstructural changes in the films, SEM was conducted to visualize the surface of prepared films.  Figure 1 shows photographs of chitosan composite films (Ch/starch + 0.5% geraniol and Ch/starch + 0.5% thymol) and SEM micrographs of the surface of the films. SEM microphotographs of the surfaces indicated a compact and homogenous structure without any large pores. A smooth, continuous structure was observed for the chitosan films surface; the presence of plasticizers caused continuities associated with the presence of geraniol or thymol in the matrix.

### 3.3. Antibacterial Activity of Chitosan Films by NB Spectrophotometric Technique

Inhibition of* A. tumefaciens*,* C. fascians*,* E. carotovora*, and* P. solanacearum in vitro* with chitosan films enriched with geraniol or thymol by NB spectrophotometric technique is shown in Figure 2. Geraniol and thymol exhibited antibacterial activity against the tested bacteria and the activity is concentration-dependent. The films with 0.5% thymol showed the strongest inhibition toward all pathogens with 60.02, 73.54, 77.99, and 74.53% inhibition of bacterial growth of* A. tumefaciens*,* C. fascians*,* E. carotovora*, and* P. solanacearum*, respectively. However, Ch/starch film showed the lowest inhibition activities (15.38, 11.10, 17.51, and 21.26% for* A. tumefaciens*,* C. fascians*,* E. carotovora*, and* P. solanacearum*, resp.).

### 3.4. Antibacterial Activity of Chitosan Films Enriched with Geraniol and Thymol by Inhibition Zone Technique

Antibacterial assay of Ch/starch films incorporated with geraniol or thymol (0.1 and 0.5%) was expressed by disk diffusion method on NA plates and the results are shown in Figure 3. The figure indicates that incorporation of thymol significantly increased the activity compared to geraniol at the same concentration. The inhibition zones obtained by film with geraniol (0.5%) were 6.67, 10.67, 7.67, and 9.33 mm for* A. tumefaciens*,* C. fascians*,* E. carotovora*, and* P. solanacearum*, respectively. However, the inhibition zones caused by film with thymol (0.5%) were 12.33, 18.33, 14.33, and 16.00 mm for* A. tumefaciens*,* C. fascians*,* E. carotovora*, and* P. solanacearum*, respectively. Photograph of the* in vitro* growth of* A. tumefaciens*,* C. fascians*,* E. carotovora*, and* P. solanacearum* in NA plates incorporated with chitosan film enriched with thymol (0.5%) is also shown in Figure 4. Ch/starch film, without geraniol or thymol, served as a control to determine its potential antimicrobial effect, but we did not observe any inhibition of the tested bacteria by the control films (Figure 4). This result may refer to the fact that the inoculum in this experiment was 10^5^–10^6^ CFU, whereas other studies have used much lower inoculum (<10^2^ CFU) for similar experiments [45, 46]. Thus, the high number of bacteria may exceed the inhibition activity of chitosan. Another explanation may be in the fact that chitosan must be dissolved to act as an antimicrobial agent. It is possible that chitosan molecules were tightly bound within the film, which prevented expression of the antimicrobial action. It can be also noted that the inhibition effects of geraniol and thymol incorporated into the chitosan films were lower than those of pure thymol with chitosan solutions (Table 1). The possible reason for the decreased activity of monoterpenes incorporated into the chitosan film could be due to partial loss potential of very volatile compounds during the preparation of the film. The other reason may be due to the leakage of controlled release of active compounds from the film during incubation period.

## 4. Conclusion

The antibacterial activity of chitosan with MW ranging from 22 to 846 kDa was studied in the present work against four crop-threatening bacteria:* A. tumefaciens*,* E. carotovora*,* C. fascians*, and* P. solanacearum*. As the concentration of chitosan increased, the antibacterial effect was strengthened and the strongest antibacterial effect was exhibited by chitosan of 22 kDa (Ch1) against the four kinds of the tested bacteria. Incorporation of the most active monoterpenes (geraniol and thymol) significantly enhanced the* in vitro* activity as in solution or in chitosan films. The Ch/starch films incorporated with thymol (0.1 and 0.5%) not only significantly enhanced the antibacterial properties but also significantly reduced the WVP compared to Ch/starch alone or the films with geraniol. This conclusion is based primarily on the application of biopolymer chitosan films as coatings for perishable agricultural products in postharvest phase, which can reduce the oxidation of lipids with the films having low WVP value.

## Figures and Tables

**Figure 1:** Photographs of chitosan composite films on the left (Ch/starch + 0.5% geraniol and Ch/starch + 0.5% thymol) and SEM micrographs of the surface of the films on the right. Scale bar 1 *μ*m and magnification ×10000 for surface morphologies of the film.

**Figure 2:** The* in vitro* inhibition of* A. tumefaciens*,* C. fascians*,* E. carotovora*, and* P. solanacearum* with chitosan films enriched with 0.1 and 0.5% geraniol or thymol by NB spectrophotometric technique. Inhibition was calculated per 0.005 g film per each treatment. Ch: chitosan; G: geraniol; T: thymol.

**Figure 3:** The* in vitro* inhibition of* A. tumefaciens*,* C. fascians*,* E. carotovora*, and* P. solanacearum* on NA plates with chitosan films enriched with 0.1 and 0.5% geraniol or thymol. Plates were inoculated with 10^5^–10^6^ colony-forming units (CFU)/plate and incubated for 48 h at 37°C. The initial disc diameter was 10 mm, and the inside diameter of Petri dish was 50 mm. Ch: chitosan; G: geraniol; T: thymol.

**Figure 4:** Photograph of the* in vitro* growth of* A. tumefaciens*,* C. fascians*,* E. carotovora*, and* P. solanacearum* in NA plates incorporated with chitosan film enriched with thymol (0.5%).

**Table 1:** The *in vitro* antibacterial activity of different molecular weights of chitosan products against *A. tumefaciens*, *C. fascians*, *E. carotovora*, and* P. solanacearum* and in combination with different concentrations of geraniol and thymol by nutrient agar (NA) dilution technique.

Chitosan product	Average MW (kDa)	MIC (mg/L)											
		*A. tumefaciens*			*C. fascians*			*E. carotovora*			*P. solanacearum*		
		Ch	Ch + G	Ch + T	Ch	Ch + G	Ch + T	Ch	Ch + G	Ch + T	Ch	Ch + G	Ch + T
Ch1	22	800	275	165	900	300	45	850	250	90	600	290	120
Ch2	32	850	240	150	950	280	40	875	230	50	725	275	110
Ch3	64	875	220	125	1000	170	25	900	210	40	825	250	100
Ch4	127	900	240	100	1075	200	40	925	230	60	875	260	100
Ch5	203	950	250	175	1100	230	50	975	250	60	900	275	90
Ch6	214	975	250	200	1125	240	60	1000	250	75	925	280	50
Ch7	241	1000	250	75	1175	275	40	1025	250	75	950	285	120
Ch8	276	1050	260	200	1200	275	25	1050	260	75	975	300	120
Ch9	300	1100	260	210	1250	280	40	1150	260	85	1050	320	130
Ch10	387	1225	275	225	1350	280	50	1275	280	100	1175	340	130
Ch11	846	1300	500	275	2600	310	80	2100	300	150	1225	375	140

Ch: chitosan; G: geraniol; T: thymol.

MIC is the minimum inhibitory concentration value obtained for each microorganism.

**Table 2:** Physicochemical properties of the modified chitosan film with geraniol and thymol.

Film	Dry weight (g) ± SE	Thickness (mm) ± SE	WVP (g/m^2^·d) ± SE	Antioxidant activity	Swelling index at time (h)			
					0.5	2.5	4	24
Ch/starch	0.150^c^ ± 0.01	0.068^b^ ± 0.01	40.12 ± 8.87	0.173^a^ ± 0.01	0.85	1.36	2.14	1.15
Ch/starch + 0.1% G	0.206^b^ ± 0.01	0.104^a^ ± 0.01	48.88 ± 1.65	0.182^a^ ± 0.02	1.75	4.27	4.69	5.10
Ch/starch + 0.5% G	0.208^b^ ± 0.01	0.107^a^ ± 0.01	70.49 ± 5.48	0.186^a^ ± 0.06	1.93	4.69	4.85	5.34
Ch/starch + 0.1% T	0.217^ab^ ± 0.00	0.114^a^ ± 0.01	36.48 ± 1.53	0.188^a^ ± 0.08	3.35	3.81	3.89	3.96
Ch/starch + 0.5% T	0.231^a^ ± 0.00	0.124^a^ ± 0.01	29.76 ± 3.29	0.192^a^ ± 0.08	1.44	2.25	3.38	2.97

Ch: chitosan; G: geraniol; T: thymol.

WVP: water vapor permeability.

Antioxidant activity expressed as mg equivalents of ascorbic acid equivalent per g of film ± SE.

Different letters in the same column indicate significant differences according to the Student-Newman-Keuls (SNK) test (*P* ≤ 0.05). Values are the mean of five replicates and are given as mean ± standard error.
